# Privacy-Preserving Reversible Data Hiding for Medical Images Employing Local Rotation

**DOI:** 10.1155/2021/5709513

**Published:** 2021-07-01

**Authors:** Guo-Dong Su, Chia-Chen Lin, Chin-Chen Chang

**Affiliations:** ^1^School of Big Data and Artificial Intelligence, Fujian Polytechnic Normal University, Fuzhou 350300, China; ^2^Department of Information Engineering and Computer Science, Feng Chia University, Taichung 40724, Taiwan; ^3^Engineering Research Center for ICH Digitalization and Multi-Source Information Fusion (Fujian Polytechnic Normal University), Fujian Province University, Fuzhou 350300, China; ^4^Department of Computer Science and Information Engineering, National Chin-Yi University of Technology, Taichung 41170, Taiwan

## Abstract

As digitalization becomes more common, patients' concerns about the leakage of private information, such as electronic medical record, are increasing, and those concerns motivated this case study of secure covert communication. Therefore, in this paper, a novel reversible data hiding method based on pixel rotation is proposed for medical images. Using pixel rotation, a state mapping model is constructed to represent the payload. More specifically, many intermediate states are derived from an image block, and each of them is used to form a one-to-one mapping relationship with a specific sequence of payload bits. In addition, to ensure the visual quality of stego-medical-images, the payload bits are only concealed in the regular blocks and the other blocks are unchanged. Moreover, the smoother regular image block will be priority to be used to embed the payload to enhance the visual quality of stego-medical-image. The experimental results showed that the stego-medical-images generated by the proposed reversible data hiding method have better visual quality with an average PSNR of 47.0307 dB, which is higher than that provided by some state-of-the-art methods.

## 1. Introduction

With the rapid development of telecommunication and computer sciences, informatization and digitization have been in many fields, such as banking and healthcare, and the result is e-banking and e-healthcare. For example, doctors use e-healthcare images for diagnosis and to study how to cure diseases. In addition, the e-healthcare platform was developed to provide a secure, covert channel of communication for the exchange of information among patients, doctors, and other relevant practitioners with the aim of ensuring that patients can access better quality medical service. However, several challenges will be encountered when electronic medical records (EMRs) are transmitted and shared in e-healthcare systems. Thus, one of the key challenges is how to ensure the security of the EMRs. Usually, the cryptography-based information security technique [1, 2] is considered to be an effective solution for this concern, but the encrypted information can easily attract the attention of attackers. Thus, the researchers in this area have focused their attention on irreversible data hiding [3–5] and reversible data hiding (RDH) [6–25] in medical images, which are techniques that can provide security and avoid attracting the attention of attackers.

RDH is a technique for processing multimedia signals that aims to hide secret data, such as EMR, into the original images, resulting in stego-images, in which the data are embedded. After removing the confidential data from the stego-images, the original images can be recovered completely. Due to its reversibility, RDH has been explored and used extensively in many applications, and detailed discussions of some of these applications are presented in Section 2.

In recent years, many RDH methods have been presented for medical images to address patients' concerns about the leakage of their private data. In 2013, Huang et al. [26] expanded the histogram shifting (HS) framework-based RDH technique to medical images that have high bit depths. For each medical image block, a difference-histogram is constructed by using different values, and it is used to carry secret data. This method satisfies 6 criteria, three of which are the inclusion of a free location map and the ability to adjust both embedding capacity (EC) and peak signal-to-noise ratio (PSNR). To improve EC, Kelkar et al. [27] presented two innovative variations of the traditional HS technique. The first technique uses HS to embed the secret data into nonoverlapping image blocks, and the second technique separates images into the region of interest (ROI) and the region of noninterest (NROI), and it only embeds the secret data in NROI. Their method leaves the medical information intact and achieves a high PSNR (above 45 dB). In the method of [28], the pixel-to-block conversion technique is used to predict the interpolated pixels in the cover image. Subsequently, the EMR related data are embedded into the LSBs of the pixels in the 4 × 4 medical image block. Instead of using the pixel-to-block conversion technique, the method in [29] uses another technique, i.e., the rhombus mean interpolation technique, as an effective alternative to interpolation for the generation of the cover image to ensure the reversibility of the medical images. Both techniques obtain a high EC and acceptable quality of the stego-medical-image. As to the method in [30], Gao et al. proposed an automatic contrast enhancement algorithm to achieve larger EC and better quality of the stego-medical-images. First, given the characteristics of the medical image, ROI and NROI are separated by using an adaptable threshold detector. Then, the ROI's histogram is stretched to enlarge the EC of ROI. For NROI, the replacement of the LSBs is applied directly, if necessary, to conceal the secret data. Gao et al.'s scheme does well in EC, but there is a significant visual difference between the stego-medical-image and its original version.

To better balance the EC and the quality of the stego-medical-image, in this paper, we propose a novel RDH method based on a local pixel rotation. The main contributions of this paper are as follows:

1. Propose an RDH based on pixel rotation. Using the rotation mechanism, many intermediate states are produced and can be used to represent the payload bits. This is quite different from other RDH methods.
2. Achieve a good balance between the EC and the quality of the stego-medical-image. Compared to some recent works, the proposed RDH method has an excellent performance in both EC and PSNR.
3. Provide secure covert communication.

The rest of this paper is organized as follows. Section 2 provides a review of RDH, and the proposed RDH method is presented in Section 3. The experimental results and analyses are presented in Section 4, and Section 5 provides our conclusions.

## 2. Related Work

The focal points of RDH are (1) how to improve the payload capability of stego-images and (2) how to enhance the quality of the stego-images. However, there is a trade-off problem between the EC and the quality of the stego-images. Most common RDH methods essentially are classified into four types, i.e., (1) difference expansion-based (DE-based) techniques [6–10], (2) prediction error expansion-based (PEE-based) techniques [11–15], (3) HS-based techniques [16–20], and (4) other techniques [21–25].

It is our understanding that the first DE framework-based RDH method was put forward by Tian [6] in 2002. In his scheme, every two adjacent pixels are compared and computed to detect the difference errors, and some of them are selected for difference expansion along with secret data embedding. Alattar [7] extended difference errors into a vector that consists of *k* distinct pixels to generate more available difference values to be used for embedding data. To improve EC, Hu et al. [8] proposed a novel DE embedding algorithm based on a dynamically expandable difference search and selection mechanism, which uses both the vertical and horizontal difference errors for embedding data. To enhance the quality of stego-images, a novel, multiple-based, RDH method based on edge prediction and lossless joint photographic experts group (JPEG-LS) pixel value prediction was presented by Wu et al. [9]. This method conceals more secret data into smooth areas rather than complex areas, thereby achieving better quality stego-images. In addition, Wang et al. [10] studied a robust RDH method using significance-bit-difference expansion. This method can be used against unintentional attacks, such as image compression and sometimes unavoidable addition of random noise, which is below a certain level and does not change the content of an image.

The PEE framework-based RDH method was developed to enhance the EC. In 2004, Thodi and Rodriguez [11] explored an algorithm that uses the correlation inherent among neighboring pixels in a local image area using a predictor. Then, the secret data are inserted by expanding the prediction error values. In 2009, Tseng and Hsieh [12] presented an RDH method based on various predictors that is capable of providing a great EC without creating any noticeable distortion. Ou et al. [13] considered the correlations among the prediction errors and used them to design a pairwise prediction error expansion for embedding secret data, and their method provided a high EC [13]. In the method of [14], the joint use of the pixel-value-ordering and PEE was developed to present a high-fidelity RDH method. Earlier, Li et al. [14] also conducted block selection before embedding the payload. Hence, this method guarantees that the PSNR of the stego-image will be greater than 51.14 dB. In 2020, Chang trained the generative adversarial networks to predict bit-planes that have been used to hide secret data. This work achieved a good performance, and it clarified how deep learning can breathe new life into older RDH methods.

The aim of the HS framework-based RDH method is to embed secret data into the peak bin that has the maximum frequency in its histogram distribution. Ni et al.'s method [16] is one of the key works in HS-based RDH methods. In [16], the zero or the minimum peaks of the image's histogram are used to embed more secret data with only slight modifications of the pixels. Next, Lee et al. [17] explored the spatial correlation of natural images to generate a more appropriate histogram, i.e., the difference-histogram. Since the difference-histogram has a much higher peak-bin, it is more suitable for RDH. Hong et al.'s HS-based RDH method [18] focuses on the modification of the prediction-error histogram to create more vacant positions for embedding secret data. Their scheme achieves a good EC and guarantees the PSNR to be above 48 dB. Jia et al. [19] considered that most of the existing RDH methods do not fully take into account that the texture of natural images influences the embedding distortion. Thus, they proposed the HS-based RDH method to reduce the invalid shifting of pixels. In this way, their method provides better-quality stego images. Also, Peng et al. [20] proposed a novel HS framework-based RDH method by a specific secret data coding strategy and a multisegment left and right histogram-shifting mechanism. Experiments showed that it achieved good performance in EC and PSNR.

In this paper, we propose an RDH method using pixel rotation to improve the EC and enhance the visual quality of medical images. More specifically, we constructed the mapping relationship between the pixel sequences and the to-be-embedded bits of the payload. This is quite different from conventional RDH methods, and the details are described in Section 3.

## 3. Proposed Scheme

In this paper, we present a novel RDH method based on pixel rotation to further enhance the EC and visual quality of stego-medical-image for medical images. Our method consists mainly of two procedures, i.e., (1) the payload embedding procedure and (2) the payload extraction procedure. However, before that, the definition of state mapping and the sequence selection are introduced.

### 3.1. Definition of State Mapping

Considering that the pixel values from a local block in a medical image are either the same or similar to each other, a rotation-based state mapping mechanism is defined and later used for embedding the payload. Let us assume that a sequence derived from a local medical image block is

(1) $$\begin{array}{c} P=\left(p_{1},p_{2},\ldots ,p_{k},\ldots ,p_{K}\right), \end{array}$$

where *K* represents the total number of elements in the current sequence, and *p*_*k*_ is its *k*^th^ element, and all ranged in [0, *V*_max_]. Next, we transfer *P* into *P*′ by

(2) $$\begin{array}{c} \left[\begin{array}{c} p_{1}^{\prime }\\ p_{2}^{\prime }\\ \ldots \\ p_{k}^{\prime }\\ \ldots \\ p_{K}^{\prime } \end{array}\right]=\left[\begin{array}{c} p_{1}\\ p_{2}\\ \ldots \\ p_{k}\\ \ldots \\ p_{K} \end{array}\right]+\varepsilon \left[\begin{array}{c} e_{1}\\ e_{2}\\ \ldots \\ e_{k}\\ \ldots \\ e_{K} \end{array}\right], \end{array}$$

where *p*_*k*_′ is the *k*^th^ element of *P*′ and *ε* is a positive integer. The value of *e*_*k*_ is determined by

(3) $$\begin{array}{c} e_{k}=\left\{\begin{array}{cc} 1, & \text{if }k=\text{pos,}\\ 0, & \text{others,} \end{array}\right. \end{array}$$

where pos is the highlighted position in *P*, and it is in the range of [1, *K*].

After that, in most cases, the *p*_pos_′ is expected to be the unique maximum value in *P*′. When *P*′ is prepared, *K* distinct states Θ^*k*^(1 ≤ *k* ≤ *K*) can be derived using the left-oriented rotation. An illustration of the state mapping definition is demonstrated in Table 1. For each row, a given state, Θ^*k*^, has a unique maximum value, *p*_pos_′. In addition, for each Θ^*k*^, the *p*_pos_′ always is located at a distinct position (i.e., in the 3^rd^ column), which can be used to carry a log_2_  *K* bit payload *s*_1_. Given a pos, the value of *a* can be computed by

(4) $$\begin{array}{c} a=\left\{\begin{array}{cc} 1, & \text{if }k>\text{pos,}\\ 0, & \text{others}, \end{array}\right. \end{array}$$

where *k* varies from 1 to *K*.

To demonstrate the definition of proposed state mapping better, Table 2 gives an example of a specific case. Here, the pos is set to 4, and the initial sequence [*p*_1_′, *p*_2_′, *p*_3_′, *p*_4_′] is [20, 20, 20, 21]. First, we rotate the initial sequence, i.e., 0, 1, 2, and 3 times separately, to generate four states, i.e., Θ^1^, Θ^2^, Θ^3^ and Θ^4^. We will find, for each state, that the position, where the maximum value is located, is different from that of the other states. Therefore, each state can be used to represent a log_2_4 bit payload.

### 3.2. Sequence Selection

For a given sequence, it is not always suitable to carry the payload. Thus, we classified the sequences into four types, i.e., the regular sequence, the singular sequence, the unusable sequence, and the overflow sequence. The definitions of those four types can be described as follows:

1. Regular sequence: the sequence has a unique maximum value, and the position of the maximum value is equal to pos
2. Singular sequence: the sequence has a unique maximum value, but the position of this maximum value is not equal to pos
3. Unusable sequence: there are two or more values that are maximum in the sequence
4. Overflow sequence: the value of the pos^th^ element in sequence exceeds *V*_max_

To explain the different types of sequences clearly, examples are provided in Table 3, where the pos and *V*_max_ are set to 4 and 127, respectively.

### 3.3. Payload Embedding

For a given 8-depth *H* × *W* medical image *I*, all pixels are divided into *N* nonoverlapping image blocks with the sizes of *h* × *w*, denoted as *I*={*I*^*t*^*|*1 ≤ *t* ≤ *N*}, where *N*=(*H*/*h*) × (*W*/*w*). For simplicity, we represent *I*^*t*^=(*I*_1_^*t*^, *I*_2_^*t*^,…, *I*_*K*_^*t*^), where *K*=*h* × *w*. Before embedding the payload, we should separate all image blocks into four types according to the definition in Subsection 3.2, and the details can be described as follows:

Step 1: process *I*^*t*^ into *P*=(*p*_1_, *p*_2_,…, *p*_*k*_,…, *p*_*K*_) using
  (5) $$\begin{array}{c} p_{k}=\text{rounding}\left(\frac{I_{k}^{t}}{2}\right), \end{array}$$
where 1 ≤ *k* ≤ *K* and the function rounding() represents the rounding operation. *p*_*k*_ is ranged in [0, 127].
Step 2: given a *ε* and pos, process *P* into *P*′=(*p*_1_′, *p*_2_′,…*p*_*k*_′,…, *p*_*K*_′) using (2) and (3).
Step 3: identify the sequence *P*′ as one of four types.
Step 4: determine *I*^*t*^ as one of four types. More specifically, if *P*′ is identified as a regular sequence, the *I*^*t*^ is determined as a regular block; if *P*′ is identified as a singular sequence, the *I*^*t*^ is determined as a singular block; if *P*′ is identified as an unusable sequence, the *I*^*t*^ is determined as an unusable block; if *P*′ is identified as an overflow sequence, the *I*^*t*^ is determined as an overflow block.

Examples of the different types of image blocks are given in Figure 1, where *ε*=1 and pos = 4.

After the separation of the image blocks, all regular blocks are roughly classified into various priority levels according to the standard deviations of their corresponding *P*'s. For a given *P*′=(*p*_1_′, *p*_2_′,…*p*_*k*_′,…, *p*_*K*_^*v*^), its various priority levels, namely, *L*, are defined as

(6) $$\begin{array}{c} L=\text{rounding}\left(\sqrt{\frac{\sum_{1}^{K}{\left(p_{k}^{\prime }-{\bar{p}}^{\prime }\right)}^{2}}{K}}\right), \end{array}$$

where $\bar{p}{}^{\prime }$ is the mean of elements in *P*′. The image block with the lower value of *L* will be the priority to be used to embed the payload for the aim of enhancing the high stego-medical-image quality. It is noted that the priority level of a regular image block will be reserved perfectly before and after payload embedding. This is because the proposed rotation based embedding strategy only changes the order of elements in *P*′ rather than changing their values.

After the classification of the regular image blocks, the payload can be embedded. First, to ensure reversibility, a location map (LM) should be used to differentiate between a regular block and a singular block. This is because a regular block may be transferred into a singular block after the payload is embedded. More specifically, if an image block is identified as a regular block, we mark it with bit “1” in LM; if an image block is identified as a singular block or unusable block or overflow block, we mark it with bit “0” in LM. Then, the LM is processed further using the quadtree-based compression technique. Next, the parameters *ε*, pos, *h*, *w*, |LM| and the compressed LM are concatenated to form the auxiliary information, where |LM| is the length of the compressed LM. The detailed analysis of LM will be given in Subsection 4.2.2. For simplicity, we used 4 bits, 4 bits, 4 bits, 4 bits, and 16 bits in our experiments to store the values of *ε*, pos, *h*, *w* and |LM|, respectively. Finally, the auxiliary information was embedded into the LSB of the first 32+|LM| pixels. Certainly, before embedding the auxiliary information, the original 32+|LM| LSBs are recorded and concatenated with secret data to form the payload. The detailed procedure of embedding payload into regular blocks is described as follows:

  Step 1: count the embedding capacity by multiplying the log_2_  *K* and the number of regular blocks. If the length of the payload is equal to or less than the embedding capacity, the embedding procedure continues; otherwise, it is terminated.
  Step 2: process all regular image blocks and process them into the corresponding sequence *P*′. Calculate the priority level for each sequence *P*′ using equation [6].
  Step 3: take log_2_  *K* bits from the head of the payload and convert them into a decimal value, d*v*.
  Step 4: read in an unused sequence *P*′ with the highest priority level. Then, rotate it left d*v* times and derive the decided sequence *P*^*∗*^ where *s*_*k*_ is equal to d*v*.
  Step 5: transfer *P*^*∗*^ to the stego-image block using the inverse process of (2).
  Step 6: repeat Steps 3 to 5 until all regular blocks have been processed, or all bits in the payload have been embedded.

After that, the stego-medical-image IS embedded with payload is generated and sent to the recipient.  Figure 2 demonstrates two examples of embedding payload bits into regular blocks, where *ε*=1 and pos = 4. In Figure 2(a), the image block is [40, 41; 41, 40], and the to-be-embedded payload bits are “01.” First, we can obtain the initial sequence [20, 20, 20, 21] (see Figure 1). Since the decimal value of payload bits is d*v* = 1, so this sequence is rotated left 1 time. The rotated sequence is decided as [20, 20, 20, 21] and put back to generate the stego-image block.  Figure 2(b) illustrates the embedding of payload bits “11” into a regular image block [40, 39; 40, 40]. In the same way, the initial sequence [19, 20, 20, 21] is obtained and rotated left 3 times. The rotated result [19, 20, 20, 21] is locked and used to generate the stego-image block [42, 41; 38, 40]. Finally, the payload bits “11” are carried out.

Besides, we also can see from Figure 2 that the distortion in Figure 2(a) is small, and the distortion in Figure 2(b) is relatively large. Overall, the distortion caused by embedding payload bits into medical images using our rotation based RDH will be affected by two aspects: (1) the more complex the image block is, the larger the distortion is; on the contrary, the smoother the image block is, the smaller the distortion is; (2) for the image block, whose complexities are similar or the same, the distortion is relevant to the times of rotation. Thus, in this paper, the smoother regular image block will be priority to be used to embed the payload to ensure the considerable visual quality of stego-medical-image.

### 3.4. Payload Extraction and Image Recovery

#### 3.4.1. State Mapping Definition in the Extraction Process

Assume that the initial sequence derived from the image block in a stego-medical-image is *PS*′=(*ps*_1_′, *ps*_2_′,…*ps*_*k*_′,…, *ps*_*K*_′). For simplicity, we also suppose that the *ps*_*k*_′ has the maximum value among this sequence. Next, the definition of state mapping used in the extraction process can be described as Table 4. An example of constructing the state mapping is given in Table 5, where *PS*′=[20,20,21,20] and pos = 4. Obviously, the sequence, whose position of the maximum value equals to pos, is the original sequence, and the corresponding *φ* is the to-be-extracted payload.

#### 3.4.2. Payload Extraction and Image Recovery

When the recipient holds the stego-medical-image *IS*, s/he can implement the extraction of payload and the recovery of the original medical image *I*. Firstly, s/he derives the auxiliary information from the every LSB of the front 32+|LM| pixels and parses out the parameters *ε*, pos, *h*, *w*, |LM| and the compressed LM. Using quadtree-based decompression, the location map is obtained that indicates which block is the regular one. Next, all pixels in *IS* are divided into *N* nonoverlapping image blocks with the sizes of *h* × *w*, denoted as *IS*={*IS*^*t*^*|*1 ≤ *t* ≤ *N*}, where *N*=(*H*/*h*) × (*W*/*w*). For simplicity, we represent *IS*^*t*^=(*IS*_1_^*t*^, *IS*_2_^*t*^,…, *IS*_*K*_^*t*^), where *K*=*h* × *w*. For the regular image blocks, the payload extraction and image recovery are conducted as follows:

Step 1: process every regular image block *IS*^*t*^ into *PS*=(*ps*_1_, *ps*_2_,…, *ps*_*k*_,…, *ps*_*K*_) using
  (7) $$\begin{array}{c} ps_{k}=\text{rounding}\left(\frac{IS_{k}^{t}}{2}\right), \end{array}$$
where 1 ≤ *k* ≤ *K*.
Step 2: according to the parameters *ε* and pos, process all *PS* into the corresponding sequence *PS*′ using (2) and (3).
Step 3: calculate the priority level of all sequences *PS*′ using equation [6].
Step 4: read in an unused sequence *PS*′ with highest priority level and rotate it right *φ* times, making the value of *ps*_pos_′ of a sequence its maximum value. Put this sequence back to generate the original medical image block, and convert *φ* into binary representation to form the payload bits.
Step 5: repeat Steps 1 to 4 until all regular blocks have been processed.

Finally, the payload is extracted completely, and the approximate original medical image is reconstructed. Next, the first 32+|LM| bits of payload are cut out and used to replace the LSB of the front 32+|LM| pixels in this approximate original medical image. By now, the secret data has been gained, and the original medical image has been recovered in a lossless way. For ease of understanding, two examples of extracting the payload bits and recovering the image blocks are illustrated in Figure 3.

## 4. Experimental Results

In this section, the results of extensive experiments are provided to evaluate the performance of the proposed RDH method. There are six 512 × 512 medical images, i.e., “Kindey_A,” “Kindey_B,” “Brain_A,” “Brain_B,” “Sketeton_A,” and “Sketeton_B,” used as test images, and they are shown in Figure 4. In our experiments, several statistical metrics, such as PSNR (Peak signal-to-noise ratio) [31] and EC, are measured for the performance evaluation.

PSNR is a metric that can evaluate the visual quality of the stego-medical-image, and it is defined as

(8) $$\begin{array}{c} \text{PSNR}=10\times \;\log_{10}\left(\frac{255\times H\times W}{\sum_{r=1}^{H}\sum_{c=1}^{W}{\left(I_{r,c}-IS_{r,c}\right)}^{2}}\right), \end{array}$$

where *I*_*r*,*c*_ and *IS*_*r*,*c*_ are the pixel values that are located on the *r*^th^ row and *c*^th^ column in images *I* and *IS*, respectively. In general, the higher the value of PSNR is, the better the visual quality of the stego-medical-image is.

EC is a metric that is used to evaluate the ability of the stego-medical-image to carry secret data, and it is defined as follows:

(9) $$\begin{array}{c} \text{EC}=\frac{H\times W}{h\times w}\times \log_{2}\left(h\times w\right),\\ \text{pure EC}=\text{EC}-\left(\left|\text{LM}\right|+32\right). \end{array}$$

### 4.1. Security Analysis

To prove that the proposed RDH method can provide the imperceptibility of secret data and stego-medical-image, security analyses, including pixel value difference (PVD) histogram [32], Shannon entropy, the number of pixels change rate (NPCR) [33], and the unified average changing intensity (UCAI) [33], were used to evaluate the stego-medical-image with full payload under *ε*=1, pos = 4, *h* = 2 and *w* = 2.

#### 4.1.1. PVD Histogram

The PVD histogram is an indicator that can provide the degree of difference between every two adjacent pixels in an image. Generally speaking, the spatially anomalous distribution of the PVD histogram leaks the existence of secret data, and it even can be used to get a rough estimation of the amount of secret data.  Figure 5 illustrates the variation tendency of the PVD histogram curves for six couples of images. As can be seen, the gaps of the PVD histogram curves between the original image, *I*, and its corresponding stego-image, *IS*, are close to each other, which implies that the proposed RDH method can resist the steganalysis of the PVD histogram.

#### 4.1.2. Shannon Entropy

Shannon entropy is a metric that can be used to evaluate the divergence of a stego-image from its original version. Generally speaking, two images coincide if their Shannon entropies are close to each other, and the system is considered to be perfectly secure.  Figure 6 shows the Shannon entropy curves of the image *I* and the stego-image *IS*, where image *IS* is embedded with different amounts of the payload. It is easy to observe that the gaps for the curves between the images *I* and *IS* are extremely close to each other. Thus, it was concluded that the proposed RDH method is extremely secure.

#### 4.1.3. Differential Attack Analysis

In addition, two measurements, i.e., NPCR and UACI, are used to provide a quantitative analysis with respect to the changes from the original image to the stego-image. NPCR is used to determine the rate at which the pixels changed for a stego-image caused by payload embedding, and it has the maximum theoretical value of 1. UACI is used to indicate the average intensity of the change of pixel values, and it has a theoretical value of 0.3346. The smaller the NPCR and UACI are, the slighter the changes in the pixel are. The UACI and NPCR are defined as follows:

(10) $$\begin{array}{c} \text{UACI}=\frac{1}{H\times W}\times \sum_{r=1}^{H}\sum_{c=1}^{W}\frac{\left|I_{r,c}-IS_{r,c}\right|}{255}\times 100\%,\\ \text{NPCR}=\frac{1}{H\times W}\times \sum_{r=1}^{H}\sum_{c=1}^{W}D_{r,c}\times 100\%,\\ D_{r,c}=\left\{\begin{array}{cc} 0, & i\text{f }I_{r,c}=IS_{r,c},\\ 1, & \text{otherwise.} \end{array}\right. \end{array}$$

Figure 7 shows the variation tendency of curves of NPCR and UACI for the stego-images that are produced for six medical images under various ECs when *ε* is set to range from 1 to 4. Obviously, in most cases, the UACI and NPCR values of the six test images are far away from their theoretical maximum values. This indicates that the proposed RDH method can effectively against differential attacks.

### 4.2. Performance Analysis

In this section, the proposed RDH method is analyzed based on its performance in terms of PSNR and EC. In these experiments, the parameters *ε*=1, pos = 4, *h* = 2 and *w* = 2 are the default values unless specified elsewhere.

#### 4.2.1. Visual Quality of the Stego-Images

After embedding the payload into the original medical image, it is always expected that the stego-image is the same or similar to the original version.  Figure 8 shows six stego-images when the EC of 60000 bits is achieved. It is obvious that the visual quality of six stego-medical-images is good, and it is difficult for the human eyes to distinguish the stego-medical-images from the original medical images.

#### 4.2.2. Analysis of LM

As analyzed in Subsection 3.3, the LM is used to differentiate the type of each image block. Because most image blocks in an image will be identified as the regular block, thus, it is expected that the LM is a sparse matrix, which can be effectively compressed into the reduced version with fewer bits.  Table 6 gives the ratio of the regular block and the size of |LM| with/without compression for six medical images. As can be seen, the ratio of the regular block reaches 76.0801% on average. What is more, the size of |LM| can be reduced from 65535 bits to 24240.67 bits. This positively contributes to achieve a high embedding capacity.

#### 4.2.3. PSNR and EC

Commonly, it is considered that it is difficult for the human vision system to detect the distortion in images, as long as the PSNR is greater than 30 dB.  Figure 9 demonstrates the graphs in terms of PSNR and EC for six images when *ε* varies from 1 to 4. It can be seen that the proposed RDH scheme can achieve a good EC that exceeds 10 × 10^4^ bits. Also, it is not surprising that the PSNR decreases as EC increases since the more payload bits are embedded onto the stego-medical-image. In addition, since the more regular blocks can be used to carry payload bits, it can be seen that the EC increases as *ε* increases. However, for a given EC, the PSNR obviously decreases when the value of *ε* is large. This is mainly due to the fact that the larger value of *ε* that is selected will lead to significant changes in pixel values during the procedure of embedding the payload.

Also, we conducted experiments using six medical images to determine the trends of PSNR and EC when the value of pos was set from 1 to 4, and Figure 10 shows the results. Figure 10 clearly indicates that, in some cases, both the trend of the PSNR curves and EC are almost consistent with each other for different values of pos. The details in the difference of PSNR are demonstrated in the subgraph embedded inside Figure 10. For images “Brain_A” and “Brain_B,” the PSNR values obtained under pos = 4 were a little lower than the values of the others, as shown in the front part of the curve. But, in general, the EC gained under pos = 4 is much higher than that of other cases. Thus, in most of our experiments, the pos = 4 is selected to achieve a good performance.

In addition, Table 7 lists the pure ECs and PSNRs obtained on six medical images for different sizes of blocks. In theory, the larger the size of the block is, the more bits the block carries. However, when the size of the block is 4 × 4, the mean value of pure EC was around 29110 bits, which was much lower than that of other cases, in which the types of block size were 4 × 4, 4 × 1, and 1 × 4. This occurred because the elements within a sequence derived from an image block are not so quite similar to each other when the block size is larger, and this leads to a serious decrement of the number of the regular blocks. In addition, it is interesting to note that, for a similar block size, the pure EC obtained for the 4 × 1 block was about 13000 bits higher than the pure EC obtained for the 1 × 4 block. That is to say, the pure EC and PSNR will be affected by the different sizes of the blocks. For example, in our experiments, the means of pure EC and PSNR reached the highest values, i.e., 75479 bits and 36.4917 dB, respectively, when the size of the block was set to 2 × 2.

### 4.3. Performance Comparison

In this section, we compare the results provided by the proposed RDH method, Parah et al.'s method [28], Geetha et al.'s method [29], and Gao et al.'s method [30] to demonstrate the excellent performance of our approach.

First, a comparison in terms of PSNR between methods [28–30] and the proposed RDH method was conducted on the six medical images that are listed in Table 8. For the sake of fairness, Table 8 gives the PSNR provided by the above four methods under the EC of 50,000 bits. It can be observed that the proposed RDH method obtains a higher PSNR than that of Parah et al.'s method [28], Geetha et al.'s method [29], and Gao et al.'s method [30], and the differences were about 18.4055 dB, 12.1389 dB, and 10.4440 dB, respectively. The main reasons are that, in the front two methods [28, 29], the use of the pixel to block technique seriously degraded the quality of the images, and, in the last method [30], the large scale in shifting pixels in order to enhance the contrast in the image leads to a decrement in the quality of the image. Also, it can be seen that the algorithm designed by Gao et al. [30] was not effective for the four images, i.e., “Kindey_A,” “Kindey_B,” “Sketeton_A,” and “Sketeton_B,” so they are marked as “NA”.

For this, we used the proposed RDH methods and methods [28, 29] on the “Brain01” and “Xray” images used in Gao et al. [30] to further evaluate their performances, and the results are presented in Figure 11. For the EC aspect, the proposed RDH method was slightly inferior compared to the other methods [28–30]. However, it was apparent that the proposed RDH scheme also achieved a considerable PSNR value, which was better than those of the other three methods [28–30] in most cases.

Secondly, comparisons of the various features of the different RDH methods are given in Table 9. In methods of [28, 29], the pixel to block conversion technique and the rhombus mean interpolation technique were used as effective means to interpolate an original medical image to a cover medical image, respectively. Then, the secret data was inserted into the LSBs of the pixels in this cover medical image to ensure its reversibility. Both of these methods can extract secret data without errors. In addition, they can reconstruct the cover medical image (but not the original medical image) in a lossless way, which was quite different from method [30] and our RDH method. Not only that, the visual quality of stego-medical-image provided by methods [28, 29] was relatively lower than that of the proposed method. Concerning the method in [30], the traditional histogram shifting technique was used to hide secret data into pixels that have peak-bin. An automatic histogram stretching technique was designed to vacate a more embeddable room. In other words, the method in [30] obtains more EC at the expense of an apparent decrease in the visual quality of stego-medical-images. It is important to note that this method has the feature of reversibility if the replacement of the LSBs is not conducted for its NROI. The proposed RDH method employs the idea of pixel rotation to insert the secret data into the medical image with reversibility. More specifically, the payload bits are carried by a specific sequence generated from a regular image block, instead of changes in the pixel values. Therefore, the proposed RDH method has a considerable PSNR of stego-medical-image.

## 5. Conclusions

In this paper, a novel rotation based RDH method for medical images is presented.

According to the characteristic of pixel distribution of the medical image, the proposed RDH method separates all image blocks into the regular blocks, singular blocks, unusable blocks, and overflow blocks. The payload is only inserted into the regular blocks to reduce the invalid rotation on pixels. Additionally, different from the conventional RDH method, we define a state mapping model to construct a mapping between various states of an image block and the payload in a one-one manner. Then, the selected state is put back into the original medical image block to form the stego-medical-image, and the payload is carried. We implemented the proposed RDH method and evaluated it with extensive experiments. It was demonstrated that our rotation based RDH method can achieve excellent performance, exceeding the performance of some recent works in both EC and PSNR. In the future, we plan to investigate the improvement of our algorithm by further considering the ROI and NORI to optimize the visual quality of stego-medical-images.

## Figures and Tables

**Figure 1:** Examples of the different types of image blocks (*ε*=1 and pos = 4).

**Figure 2:** Examples of embedding payload bits into regular blocks (*ε*=1 and pos = 4).

**Figure 3:** Examples of extracting the payload bits and recovering the image blocks (*ε*=1 and pos = 4).

**Figure 4:** Six test medical images. (a) Kidney_A; (b) Kidney_B; (c) Brain_A; (d) Brain_B; (e) Sketeton_A; (f) Sketeton_B.

**Figure 5:** Six PVD histograms of images (I) and *IS*. (a) Kidney_A; (b) Kidney_A; (c) Brain_A; (d) Brain_B; (e) Sketeton_A; (f) Sketeton_B.

**Figure 6:** Shannon entropy curves of images (I) and *IS*. (a) Kidney_A; (b) Kidney_B; (c) Brain_A; (d) Brain_B; (e) Sketeton_A; (f) Sketeton_B.

**Figure 7:** Curves of NPRC and UACI for the stego-images. (a) NPRC. (b) UACI.

**Figure 8:** Stego-medical-images: (a) Kidney_A; (b) Kidney_B; (c) Brain_A; (d) Brain_B; (e) Sketeton_A; (f) Sketeton_B.

**Figure 9:** Graphs in terms of PSNR and EC for six medical images when *ε* varies from 1 to 4. (a) Kidney_A; (b) Kidney_B; (c) Brain_A; (d) Brain_B; (e) Sketeton_A; (f) Sketeton_B.

**Figure 10:** Graphs in terms of PSNR and EC for six medical images where pos varies from 1 to 4. (a) Kidney_A; (b) Kidney_B; (c) Brain_A; (d) Brain_B; (e) Sketeton_A; (f) Sketeton_B.

**Figure 11:** Graphs showing the PSNR and EC values for two medical images. (a) “Brain01”; (b) “Xray”.

**Table 1:** Illustration of the state mapping definition (rotation left).

	States Θ^*k*^(1 ≤ *k* ≤ *K*)	Position of maximum value	Payload *s*_1_
Θ^1^	[*p*_1_′, *p*_2_′,…, *p*_pos_′,…, *p*_*K*_′]	pos + *K a*	0
Θ^2^	[*p*_2_′,…, *p*_pos_′,…, *p*_*K*_′, *p*_1_′]	pos − 1 + *K a*	1
…			
Θ^*k*^	[*p*_*k*_′,…, *p*_pos_′,…, *p*_*K*_′, *p*_1_′,…, *p*_*K*−1_′]	pos − (*k* − 1) + *K a*	*k* − 1
…			
Θ^*K*^	[*p*_*K*_′, *p*_1_′, *p*_2_′ …, *p*_pos_′,…, *p*_*K*−1_′]	pos − (*K* − 1) + *K a*	*K* − 1

**Table 2:** An example of constructing the state mapping.

	States Θ^*k*^	Position of *p*_pos_′	Payload *s*_1_
Θ^1^	[20,20,20,21]	4	0
Θ^2^	[20,20,21,20]	3	1
Θ^3^	[20,21,20,20]	2	2
Θ^4^	[21,20,20,20]	1	3

**Table 3:** Examples of different types of sequences (pos = 4).

Sequences	Situations	Block types
[20,20,20,21]	*p*_pos_′=*p*_4_′ is unique maximum value	Regular
[20,20,21,20]	*p*_pos_′=*p*_4_′ is not unique maximum value	Singular
[20,19,20,21]	*p*_pos_′=*p*_4_′ is unique maximum value	Regular
[20,20,21,21]	*p*_pos_′=*p*_4_′ is not unique maximum value	Unusable
[127,127,126,128]	*p*_pos_′=*p*_4_′=128 > *V*_max_=127	Overflow

**Table 4:** Illustration of the state mapping definition used in extraction process (rotation right).

	States Θ^*k*^(1 ≤ *k* ≤ *K*)	Position of maximum value	Payload *s*_1_
Θ^1^	[*ps*_1_′, *ps*_2_′,…, *ps*_*k*_′,…, *ps*_*K*_′]	*k*	0
Θ^2^	[*ps*_*K*_′, *ps*_1_′, *ps*_2_′,…, *ps*_*k*_′,…, *ps*_*K*−1_′]	*k*+1	1
…			
Θ^*k*^	[*p*_*k*_′,…, *p*_pos_′,…, *p*_*K*_′, *p*_1_′,…, *p*_*k*−1_′]	pos	*φ*
…			
Θ^*K*^	[*p*_*K*_′, *p*_1_′, *p*_2_′ …, *p*_pos_′,…, *p*_*K*−1_′]	*k* − 1	*K* − 1

**Table 5:** An example of constructing the state mapping used in extraction process (rotation right).

	States Θ^*k*^	Position of maximum value	Payload *s*_1_
Θ^1^	[20,20,21,20]	Payload *s*_1_	0
Θ^2^	[20,20,20,21]	4 (pos)	1 (*φ*)
Θ^3^	[21,20,20,20]	1	2
Θ^4^	[20,21,20,20]	2	3

**Table 6:** Size of the |LM| and ratio of the regular block for six medical images

	|LM| without compression	|LM| with compression	Ratio of regular block (%)
Kidney_A	65536 bits	20898 bits	82.2159
Kidney_B	65536 bits	38756 bits	67.9978
Brain_A	65536 bits	16429 bits	84.8206
Brain_B	65536 bits	33596 bits	71.0617
Sketeton_A	65536 bits	22077 bits	71.0022
Sketeton_B	65536 bits	13688 bits	79.3823
**Average**	**65536** bits	**24240.67**	**76.0801**

**Table 7:** Pure ECs (bits) and PSNRs (dB) obtained on six medical images with different block sizes.

Images	Block size (unit: pixels)							
	2 × 2		4 × 1		1 × 4		4 × 4	
	Pure EC	PSNR	Pure EC	PSNR	Pure EC	PSNR	Pure EC	PSNR
Kidney_A	86864	34.6457	86755	28.5421	79886	31.7735	42777	31.3795
Kidney_B	50370	31.2902	50756	26.3472	37386	28.2342	27379	30.1879
Brain_A	94747	36.1669	71924	30.9600	62540	32.7430	7151	33.2414
Brain_B	59546	34.3169	41513	30.7882	34905	29.9029	NA	NA
Sketeton_A	70987	39.9571	79830	39.73034	55944	32.9566	25352	36.7719
Sketeton_B	90360	42.5736	92830	41.0707	81843	37.1164	42889	38.2895
**Average**	**75479**	**36.4917**	**70601**	**32.9064**	**58751**	**32.1211**	**29110**	**33.9740**

NA: Not applicable.

**Table 8:** Comparisons of PSNRs for different RDH methods under the EC of 50,000 bits.

Images	PSNRs (dB)			
	Parah et al. [28]	Geetha et al. [29]	Gao et al. [30]	Proposed method
Kidney_A	28.6677	34.4016	NA	52.0954
Kidney_B	24.4430	28.5094	NA	51.5742
Brain_A	32.6299	39.3391	39.8084	48.4490
Brain_B	30.1521	36.1370	38.2170	46.9342
Sketeton_A	35.3404	42.6602	NA	49.5485
Sketeton_B	38.0766	45.8597	NA	51.1387
**Average**	**31.5512**	**37.8178**	**39.5127**	**49.9567**

NA: not applicable.

**Table 9:** Comparisons of features for different RDH methods.

Features	Parah et al. [28]	Geetha et al. [29]	Gao et al. [30]	Proposed method
Methodology	Pixel to block technique	Rhombus mean interpolation technique	Histogram shifting	Pixels rotation
Hidden component	LSBs	LSBs	Pixels	Pixels
Bit errors	No	No	No	No
PSNR (on average)	−(30.4335 dB)	(36.7489 dB)	−(29.1779 dB)	(47.0307 dB)
Reversibility	No	No	Yes	Yes

More “+” means better image quality when compared to the Refs. [28, 30]. The symbol “−” represents the baseline in terms of PSNR.

## Data Availability

All the data can be accessed in the public database.
